# Influence of Aerobic Exercise Load Intensity on Children's Mental Health

This article has been retracted.

**DOI:** 10.1155/2022/7827980

**Published:** 2022-06-11

**Authors:** Sihong Zhao

**Affiliations:** School of Preschool Education, Xi'an University, Xi'an 710065, Shaanxi, China

## Abstract

As people have become more aware in recent years, aerobic physical exercise plays an important role in alleviating people's mental health problems. However, traditionally, it is believed that young children do not have mental health problems. To help people change this fixed idea, and to study how to correctly adjust the load intensity of aerobic physical exercise under the condition of limited physical fitness of young children, and accurately help children's mental health development, this paper studies the influence of aerobic physical exercise load intensity on children's mental health. In this paper, the detection and tracking technology of video moving objects is used to analyze the data of the research object. This technique includes several commonly used and improved video analysis algorithms. The use of moving target and tracking technology and algorithms can completely extract moving targets, eliminate the phenomenon of void and nothingness, and improve data acquisition and analysis capabilities. The results show that taking part in aerobic exercise with appropriate intensity is beneficial to regulating children's emotional state, reducing their psychological burden, enhancing their negative energy resistance, and arousing their positive participation. Compared with before aerobic exercise, the learning efficiency was improved by 6.36%.

## 1. Introduction

Children's mental health of the mental is the focus of increasing social concern. Children's mental health of mental is an important prerequisite for preschool education. Preschool education is the foundation of the national quality education system, which can lay a good foundation for children's future life and provide them with good development conditions. Therefore, it is more important and urgent to actively explore the relationship between aerobic exercise load intensity and children's health, and the influence of physical exercise activities on children's mental health and positive results.

Aerobic exercise is a key part of physical exercise and plays a heavy role in enhancing students' physical fitness. Many teams have studied this. Gregory team studied the effects of dual-task gait training and aerobic exercise intervention on cognition. It investigated the activity and cardiovascular health of elderly people living in a community without dementia. The conclusion is that aerobic exercise improves the performance of many cognitive results [1]. Several studies by Innocenti have shown that aerobic exercise can improve the cognitive ability of MCI patients [2]. Chan studied that exercise training can improve insulin sensitivity and RBP4 [3]. The purpose of Callegari's research was to investigate the muscle response of creatine kinase (CK) and lactate dehydrogenase (LDH) after different levels of resistance and aerobic exercise programs. Immediately after the end of the protocol, it was observed that LDH in some groups increased significantly compared with other groups [4]. The AJA team tested whether Mk III GLCS was the second largest aerobic exercise. The feasible auxiliary means of VO_2_ max prediction produced by this method is to compare the obtained VO_2_ max prediction with pa [5]. Leeuwis had evidence that aerobic exercise is beneficial to cognition and provided insight into the potential mechanisms of aerobic exercise in improving hemodynamic status [6]. The research by Moghadasi indicated that high-intensity aerobic exercise training greatly affected serum A-FABP [7]. The results of these studies show that aerobic exercise plays an essential role in the human body.

In the process of children's development, it is important to pay attention to their physical and mental health. Considering children's health, it should not only consider the healthy development of young children. Children's mental health is related to their healthy development in the future. Caring for children's mental health means paying attention to children's healthy development. Many teams have studied this. Freeman's research held that psychological health problems are intimately related to the environment [8]. Silove considered the contemporary problems in the field of refugee mental health. He discussed developing ecological research model focusing on the dynamic relationship among past traumatic experiences, continuous daily stressors, and background destruction of the core social psychological system [9]. Butterworth's research has shown that adolescents and young people have high psychological stress, but the utilization rate of treatment is very low [10]. Emma studied and compared parents' and children's reports on children's mental health to determine the relationship between parent-child differences and parents' psychological and attitude factors, and how parent-child differences are related to the use of professional services [11]. Leese measured different types of service provision and considered that the influence on the views of service users was essential for planning mental health services [12]. Based on the PREPARE/ENRICH program, Muhammad found the influence of communication and conflict resolution skills training on the mental health of Iranian couples [13]. Tsanava believed that early intervention for children and adolescents with mental health problems is essential to ensure that these problems will not continue into adulthood [14]. The results have shown that it is essential to solve children's mental health problems, which will have an important impact on their future.

The points of innovation in this document are as follows:

1. In the field of aerobic psychology, experienced experts and researchers have done a great deal of research and different degrees of research on the effects of exercise on health. In addition, there is no uniform standard for training intensity, duration, and frequency.
2. According to children's age, under the condition that the same exercise cycle, the same number of exercises per week, and intensity are close to three emotional factors, the topics are grouped into three types of functions. It is an exercise plan to analyze each mental health level. It adjusts the relationship between different physical activities and mental health plans according to different mental health levels and provides some clues for the influence of different physical activity plans on mental health.
3. This work is the first time to use the human motion search and tracking system, which uses a video imaging algorithm to study the influence of aerobic exercise weight on children's mental health. It improves the efficiency of data analysis, ensures the accuracy of the data, and provides a new basis for future research.

## 2. Methods

The research focus of this paper is to detect and track aerobic exercise videos, which needs to gather and parse a large amount of data. To facilitate data analysis, this paper uses a new video processing algorithm to help obtain and process data on the relationship between young children and physical exercise load intensity. It simplifies the extracted image to reduce the interference elements of key algorithms in the later stage, including the subsequent processes and algorithms [15].

### 2.1. Gray-Scale Processing

Color images are divided into three categories: black and white, gray, and color. The natural video images taken by digital cameras are all color images. To speed up the program, it is important to convert the downloaded image into a gray image. Gray scale can represent the total area and distribution area of the whole image as well as the color and brightness characteristics [16].

The relationship usually adopts the formula:

(1) $$\begin{array}{c} grey\left(x,y\right)=0.\;11r\left(x,y\right)+0.59\left(x,y\right)+0.3b\left(x,y\right). \end{array}$$

### 2.2. Image Enhancement Algorithms

Image enhancement technology can increase users' interest in images, such as edges, borders, and contrast, and increase the contrast between different parts of images [17]. It can provide a good foundation for extracting image information and applying other analysis techniques. Improving image information, lighting and shadow, and sharpening image edges are the main concerns of image enhancement. Gray-scale conversion technology is an important way to enhance the effect of image recognition, which makes the details of the image easy to find.

(2) $$\begin{array}{c} S=T\left(r\right). \end{array}$$

Among them, *r* and *s* represent the image pixel values before and after processing. It is a transformation method that maps the original domain *r*_*o*_, *r*_*k*_ to the latest domain *S*_*o*_, *S*_*k*_.

Different interpretations of *t* may lead to different conversion results. Typical gray-scale modification includes linear inversion transformation, logarithmic transformation, contrast rendering, and histogram alignment.

(1) Contrast stretching:

(3) $$\begin{array}{c} s=T\left(r\right)=\frac{1}{1+\left(m/r\right)E}. \end{array}$$

Among them, E is a given parameter of control degree and M is the maximum value of the gray scale. Histogram averaging changes the input gray level according to the formula (x, x) [18] to obtain the gray output level *s*.

(4) $$\begin{array}{c} s=E\left(a\right)=\int \begin{array}{c} 1\\ 0 \end{array}P_{a}\left(u\right)\text{d}u. \end{array}$$

In the above formula, *pa*(*u*) represents the probability density function of the gray level in a given image and *w* is the variable of sum. Next, it can be assumed that the probability weight function of the bright gray scale is uniform, that is:

(5) $$\begin{array}{c} p_{a}\left(a\right)=\left\{\begin{array}{cc} 1, & 0\leq a\leq 1\\ 0, & \text{others} \end{array}.\right. \end{array}$$

After histogram adjustment, the gray scale is more balanced, and the final image has higher contrast and wider intensity.

(2) Two-dimensional median filtering: in a digital image, because it is a 2-dimensional data image, the intermediate processing is also 2-dimensional. It selects a 2-dimensional recording model with specific settings. The process of presenting the 2D filter is as follows:

(6) $$\begin{array}{c} h\left(x,y\right)=\text{Med}f\left(x-u,y-v\right),\;\left(u,v\right)\in D. \end{array}$$

Among them, *f*(*x*, *y*) is the original image, *h*(*x*, *y*) is the median filtered image, and D is the two-dimensional template.

(3) Mean filtering: assuming that the size of video *f*(*x*, *y*) with noise is *M∗N*. The formula of processed image $\tilde{f}\left(i,j\right)$ is as follows, where W is the domain of point (x,y).

(7) $$\begin{array}{c} \tilde{f}\left(i,j\right)=\frac{1}{M*N}\sum_{i,jeW}f\left(i,j\right). \end{array}$$

(4) Gaussian filtering: Gaussian smoothing filter is the most widely used algorithm in image processing [19].

(8) $$\begin{array}{c} f^{\prime }\left(i,j\right)*g\left(i,j\right), \end{array}$$

(9) $$\begin{array}{c} g\left(i,j\right)=\frac{1}{\sqrt{2\pi \alpha }}\exp\left(-\frac{i^{2}+j^{2}}{2\alpha^{2}}\right). \end{array}$$

Among them, *α* is the characteristic parameter of Gaussian low-pass filtering. To blur the edge of the image, so as not to affect the normal performance of the next algorithm, this effect can be achieved by adjusting the filter.

(5) Three-frame difference algorithm: the algorithm of frame difference method is simple and clear, and background update is not considered. The shortcomings are also very obvious. Difference images always have a lot of noise. To solve this problem, a three-frame difference method is proposed, and its formula is

(10) $$\begin{array}{c} mx\left(x,y\right)=\left|f_{t-1}\left(x,y\right)-f_{1}\left(x,y\right)|*\right|f_{x}\left(x,y\right)-f_{t+1}\left(x,y\right)|, \end{array}$$

(11) $$\begin{array}{c} M_{x}\left(x,y\right)=\left\{\begin{array}{c} 255,m_{x}\\ \text{0} \end{array}\right.\left(x,y\right)>T. \end{array}$$

Among them, the first frame of the three-frame difference image is *f*_*t*−1_(*x*, *y*), the second frame is *f*_*t*_(*x*, *y*), the third frame is *f*_*t*+1_(*x*, *y*), and *m*_*t*_(*x*, *y*) is the three-frame conversion part.

(6) Background subtraction method: background subtraction is the process of removing each image frame with a fixed background pattern. This is also a common algorithm for moving target detection. The expression formula is as follows:

(12) $$\begin{array}{c} R\left(x,y\right)=F\left(x,y\right)-G\left(x,y\right). \end{array}$$

Among them, *R*(*x*, *y*) is the moving target to be detected and *F*(*x*, *y*) is the video sequence image. *G*(*x*, *y*) is the background model image.

(7) Optical flow constraint method: when the recording time is *t*, the gray value of the moving object of the image in space (x, y) is E (x, *y*, and t). When it reaches the (*x*+Δ*x*, *y*+Δ*y*) point and its gray matter is recorded as *E*(*x*+Δ*x*, *y*+Δ*y*, *t*+Δ*t*), according to the constant light hypothesis, there are

(13) $$\begin{array}{c} \frac{\text{d}E}{\text{d}t}=0. \end{array}$$

According to the chain rule,

(14) $$\begin{array}{c} \frac{\partial E}{\partial x}\frac{\text{d}x}{\text{d}t}+\frac{\partial E}{\partial y}\frac{\text{d}y}{\text{d}t}+\frac{\partial E}{\partial t}=0. \end{array}$$

Marking it as *μ*=d*x*/d*t*, *υ*=dy/d*t*. It is the time of the moment projection component (x, y) in the *μ*, *υ* image plane in the *X* direction and *Y* direction, that is, the bright flux. This provides us with the linear equation of visual flow:

(15) $$\begin{array}{c} E_{x}u+E_{y}v+E_{t}=0. \end{array}$$

This is a well-known optical flow constraint equation, and the value of *E*_*x*_=∂*E*/∂*x*, *E*_*y*_=∂*E*/∂*y*, *E*_*t*_=∂*E*/∂*t* can be obtained from the image. The Laplacian operator of U and *v* is defined as follows:

(16) $$\begin{array}{c} \nabla^{2}u={\left(\frac{\partial u}{\partial x}\right)}^{2}+{\left(\frac{\partial u}{\partial y}\right)}^{2},\\ \nabla^{2}v={\left(\frac{\partial v}{\partial x}\right)}^{2}+{\left(\frac{\partial v}{\partial y}\right)}^{2}. \end{array}$$

According to the optical flow constraint equation, the error reflection of bright flux deviation from normal light is

(17) $$\begin{array}{c} \Gamma_{b}=E_{x}u+E_{y}y+E_{t}. \end{array}$$

The error of deviation from the smoothness requirement is

(18) $$\begin{array}{c} \Gamma_{e}={\left(\frac{\partial u}{\partial x}\right)}^{2}+{\left(\frac{\partial u}{\partial y}\right)}^{2}+{\left(\frac{\partial v}{\partial x}\right)}^{2}+{\left(\frac{\partial v}{\partial y}\right)}^{2}. \end{array}$$

Minimizing error:

(19) $$\begin{array}{c} \Gamma^{2}=\int \int \alpha^{2}\Gamma \begin{array}{c} 2\\ c \end{array}+\Gamma \begin{array}{c} 2\\ b \end{array},\text{d}x\text{d}xy. \end{array}$$

Solving the equation:

(20) $$\begin{array}{c} u^{n+1}=\begin{array}{c} -n\\ u \end{array}-\frac{\left[E_{x}\begin{array}{c} -n\\ u \end{array}+E_{y}\begin{array}{c} -n\\ v \end{array}+E\begin{array}{c} t \end{array}\right]}{\left(\partial^{2}+E\begin{array}{c} 2\\ x \end{array}+E\begin{array}{c} 2\\ y \end{array}\right)}, \end{array}$$

(21) $$\begin{array}{c} v^{n+1}=\begin{array}{c} -n\\ v \end{array}-\frac{E_{x}\left[E_{x}\begin{array}{c} -n\\ u \end{array}+E_{y}\begin{array}{c} -n\\ v \end{array}+E\begin{array}{c} t \end{array}\right]}{\left(\alpha^{2}+E\begin{array}{c} 2\\ X \end{array}+E\begin{array}{c} 2\\ y \end{array}\right)}. \end{array}$$

With the development of computer, Internet, and other technologies, the data processing technology of physical exercise video is also increasingly widely used in various fields. By making good use of the video processing technology and its algorithm, the data of aerobic physical exercise can be accurately obtained, the influence of the load intensity of physical exercise on the mental health of young children can be observed, and a quick response can be made. This provides a firm foundation for improving the mental health of young children.

## 3. Intelligent Surveillance and Video System

### 3.1. Intelligent Surveillance and Video Composition

By finding targets and monitoring systems [20], it collects and processes information on the effects of aerobic physical activity and load intensity, which play an important role in early childhood development and people's mental health. It analyzes and evaluates this, providing accurate data for research. Therefore, this paper uses the search sports video streaming media site and tracking system to enable the results. The main users of this program include system administrators, temporary users, and sponsors. Users use Ethernet to access the Internet and then use firewalls to connect to routers and gateways for data mining, as shown in Figure 1.

### 3.2. System Modules

(1) Physical exercise video management module: the physical exercise video control module is an important part of the search engine module. The video control module is mainly managed and maintained by video managers. Its functions mainly include video control functions and video management functions. Among them, the main function of sports video management is to maintain sports videos, including adding videos, deleting, and converting videos. [21]. The video administrator inputs the corresponding user name and password to enter the settings, then accesses the physical exercise video control module, and completes the video recovery process by prompting the video method, as show in Figure 2.

(2) Target tracking management module: the most important part of the target search and tracking system is the target tracking module. The main function of the unit is to monitor the transfer position in real time, and then retrieve the corresponding data and analyze it with the help of monitoring. The function of this part is to support children's mental health, and its primary responsibility is the video analyst. The main tasks of this project are the development of a space models and the monitoring of space events. The specific operation procedure is as follows: First, design a fixed shooting position, and then design the correct monitoring position, as shown in Figure 3.

Intelligent monitoring and video systems are mainly used in the fields of vehicle monitoring, electric energy measurement, on-site monitoring, and so on [22]. The purpose of this book is to explore the intensity of teenagers' aerobic exercise by using search and stadium tracking system, video monitoring, tracking, and stadium tracking activities. The use of intelligent monitoring and video systems to detect the impact of aerobic physical activity on child program implementation has an important and positive role in the development of children's mental health. In addition, the use of this system can also simplify the complicated data collection process and improve the research efficiency.

### 3.3. Simulation of Actual Space Scene

Figure 4 shows the actual space scene. It selects the direction OX perpendicular to the ground plane as the reference direction. HF represents the footprint to be measured. *L* is the predicted plane image of the zero line on the infinite surface. When the pedestrian stands with his feet locked, the top line of the pedestal can be approximately a part of the line perpendicular to the ground. That is, the field of vision of the head and feet, so HF is equivalent to the reference direction OZ. H0F0 represents the reference point selected in the real scene. C refers to the movement of the camera, and its vertical distance from the ground plane is represented by dc. It draws a plane parallel to the ground plane by moving the camera, and the extension line of the line segment HF intersects with the plane A at point P, so the distance from point P to the ground plane [14] is equal to dc.

## 4. Specific Methods of Aerobic Exercise

Research object: to study the influence of aerobic exercise on children's mental health, this paper selects 80 children aged 61–70 months in kindergarten and divides them into two teams. One team is the experimental team and the other team is the control team. There are 20 children in each group. The reason the kindergarten is chosen is that the children in large classes are suitable in age and easy to control process. All children who participated in the study obtained the consent and support of parents and the school in advance. In addition, before the start of the test, the test group and the control group were randomly divided into groups to conduct a preliminary mental health test at the time of group selection. The two groups of children were almost identical, which allowed the test to ignore the differences and randomly determine the experimental group and the control group of young children.

Since all children who participate in the training are young, organized training is unique to children's basic sports, but the simple content is related to aerobic exercise. It allows children in the experimental group to take part in aerobic exercise and uses unconventional aerobic exercise methods to have extra influence on the test group. Basic gymnastics for children is a simple and easy-to-operate aerobic exercise program. It compiles 3 sets of infant aerobics, supplemented by small games. Children in the control group were intervened by the high, medium, and low intensity of basic gymnastics. Each group of children participated in the same load intensity exercise for 2 months, 8 times a month, and 2 times a week, and the time of each exercise was 30 minutes. Time arrangement: one time is arranged in the physical education class, one time is arranged after class, and the control group is the same as usual. To show the intensity of aerobic exercise, it needs to apply the heart rate index. High-intensity exercise requires the heart rate to reach more than 140 beats/min, 110 ∼ 130 beats/min is suitable for the goal of medium-intensity exercise, and less than 100 beats/min is the goal of low-intensity exercise.

It tests the mental health of children. After the experiment, the children's mental health status was checked again by preventive mental health test and the results of both were carried out. At the same time, sports emotion measurement is used to measure cognitive emotion and sports satisfaction after different degrees of exercise, and make statistical analysis, as shown in Figure 5.

Control factors of the experiment: during the period, children's gymnastics basic training was used to intervene, and all training items were carried out on the plastic playground. To ensure proper physical exercise improvement and normal operation, teachers must implement the protection system. To ensure the effectiveness of exercise, the duration of each exercise is 30 minutes.

Experimental control factors: in the whole process of this study, only the trainers know the course, but the children do not know that they are the subjects. This is to prevent the Hawthorne effect of the controller from affecting the result. The Hawthorne effect refers to the artifact of the method in field behavioral experiments, as subjects realize they are being trained. This knowledge allows them to respond to the social context of the data collection process, rather than to the experimental methods the researchers are trying to investigate. It is similar to the “guinea pig effect” in laboratory studies. During the experiment, in the physical activity classes of the two classes, the experimental group carried out a well-designed basic exercise plan for children, while the control group received the contents of preschool textbooks for routine activities. Other conditions being completely equal, two groups of children were tested.

Posttreatment: after the experiment, two groups of children were tested, excluding various factors (taking part in additional training such as dancing and roller skating). Mathematical statistics: SPSS 20.0 is used for statistical calculation based on experimental data, and its related data are essential for statistical analysis. Gender analysis is used to evaluate the influence of basic sports on children's mental health in many fields.

## 5. Outcomes of Aerobic Exercise Experiment

### 5.1. Comparison of Mental Health Status of Children in Experimental Group and Control Group before Exercise

(1) Before the experiment, the health level of the students in the experimental class, the control class, and the research class in aspects of insight, intelligence, emotional experience, sense of responsibility, thinking, language, anxiety level, self-esteem, self-confidence, and memory was checked. Physical exercise experiments are based on differences, as shown in Figure 6.

From Figure 6, the average success rate of children's mental health in the experimental group is 70.04%, and that of girls is 69.51%. The average pass rate of boys in the control group and the mental health of children in the experimental group reached 70.62%, and the average of the two groups was 70.61%. There is no significant age difference, and they are at the same level.

In addition, it can be seen from Figure 6 that there is no significant difference in the mental health level between the experimental group and the control group before the experiment, which can be related and studied. The data thus obtained is more reliable.

### 5.2. Comparison of Mental Health Status between Experimental Group and Control Group before the Experiment

As can be seen from Figure 7, before the experiment, we analyzed the test results of several indexes of children's mental health in the experimental group and the control group and found that there was no significant difference in each index. The experimental group is almost the same as the control group. The experiment can begin formally.

### 5.3. Comparison of Mental Health Status of Postnatal Children

The students were tested and investigated in aspects of mental health level, insight, intelligence, emotional experience, sense of responsibility, thinking, language, anxiety level, self-esteem and self-confidence, memory, etc.

To make the data clearer, the numerical values are averaged and expressed by *P*^*∗*^100. When *P*^*∗*^100 < 5, the difference is significant; *P*^*∗*^100 < 1, the difference is highly significant. When *P*^*∗*^100 > 5, there was no significant difference.

From the data in Figure 8, it can be seen that there are differences in the scores of insight, intelligence, emotional experience, sense of responsibility, thinking, language, anxiety level, self-esteem, and self-confidence and memory during the whole experiment (*P*^*∗*^100 − 5). Comparing the mental health level of the experimental group and the control group, the growth rate of different positions is different. Comparing the increase of scores before and after, it is concluded that there are significant differences in intelligence and thinking. The scores of self-esteem and anxiety levels are not as obvious as those of other parts, and there are obvious changes in language and emotional experience. During the whole experiment, the sense of responsibility and memory scores will increase rapidly.

### 5.4. Comparison of Mental Health Indexes of Children in Experimental Group and Control Group before and after Treatment

After the experiment, it is necessary to compare and analyze the data obtained from the control group and the experimental group, as shown in Figure 9.

As can be seen from Figure 9, after children's basic gymnastics training, there are significant differences in the mental health categories of children in the experimental group, such as insight, intelligence, emotional experience, sense of responsibility, thinking, language, anxiety level, self-esteem and self-confidence, and memory. (*P*^*∗*^100 < 5). Among them, the scores of thinking and language in the experimental group are quite different. The scores of intelligence, emotional experience, and anxiety level vary greatly. By comparing the scores of the mental health test report of the experimental group before and after the test, the average scores of several modules have been significantly improved, which shows that children's basic gymnastics has a significant impact on the improvement. In addition, from Figure 9, it can be found that there is no significant difference in the scores of several aspects of children's mental health in the control group (*P*^*∗*^100 − 5), but the overall trend score increases. The mental health level of children in the control class has no basic exercise. Each specific part changes at a different speed under the intervention.

## 6. Discussion and Conclusions

### 6.1. Discussion

Through this study, the following results are obtained:

1. Participating in aerobic exercise of appropriate intensity is helpful to regulate children's emotional state and enhance their mental health. It is necessary to renew ideas, reduce children's learning burden and homework, guide them to actively participate in physical exercise, and cultivate their interest and behavior in physical exercise, to lay a solid foundation for life sports.
2. Children from 65 to 70 months participating in high- and medium-intensity aerobic exercise can achieve greater psychological effects of exercise and more pleasure in exercise. From 61 to 65 months, children participating in moderate and low-intensity aerobic exercise can achieve greater psychological effects of exercise and more pleasure in exercise. 61–65 months of young children participating in high-intensity exercise did not benefit their mental health.
3. There were no gender differences in children participating in different intensities of aerobic exercise. The development of children's aerobic exercise programs should take into account physical, psychological, age and gender and other factors.

### 6.2. Conclusion

To study the influence of aerobic exercise and its load intensity on children's mental health, this paper adopts the classical pedestrian detection algorithm. It detects pedestrians in every frame of the video in this paper. There are more than 140 frames in the video, and the detection accuracy is 89%. It successfully detects the human body in the moving window. Detecting the human body in the moving area saves a lot of calculation time compared to detecting the whole picture. However, the accuracy rate has declined to some extent, which is related to the size of the training samples. It fills the moving window to make it regular, so that it can be used for detection. It zooms in and out during detection and makes multiscale detection more accurate. Finally, aiming at the multiwindow fusion problem caused by multiscale detection, the local MeanShift method is adopted to fuse, which ensures the fusion effect and effectively avoids the problem of fusing multiple human bodies into one window.

To further study the influence of children's basic gymnastics on children's mental health, this study conducted in-depth research on children's cognition, emotion, and social interaction. Through this study, it is found that children's scores in all aspects of mental health will gradually increase with the increase of age, and the change speed of each specific aspect is different. Aerobic exercise can effectively improve children's mental health. Compared with the control group, there is a highly significant difference in the movement of children who take part in aerobic exercise. This shows that aerobic physical exercise can promote the healthy development of children's mental health. Children's aerobic exercise can be included in kindergarten teaching materials as one of the educational means of all-round development, so that it can develop along the scientific direction.

## Figures and Tables

**Figure 1:** System information collection diagram.

**Figure 2:** Physical exercise video management module diagram.

**Figure 3:** Target tracking management chart.

**Figure 4:** Simulation diagram of actual space.

**Figure 5:** Flow chart.

**Figure 6:** Qualified of children's mental health.

**Figure 7:** Comparison of mental health status between experimental group and control group before the experiment.

**Figure 8:** Statistical table of children's mental health in experimental group and control group experiment.

**Figure 9:** Comparative analysis of children's mental health level between experimental group and control group before and after the experiment.

## Data Availability

All the data used are included in the article.
